RETRACTED

# Second-Generation Histamine H1 Receptor Antagonists Suppress Delayed Rectifier K^+^-Channel Currents in Murine Thymocytes

**DOI:** 10.1155/2019/6261951

**Published:** 2019-04-30

**Authors:** Kazutomo Saito, Nozomu Abe, Hiroaki Toyama, Yutaka Ejima, Masanori Yamauchi, Hajime Mushiake, Itsuro Kazama

**Affiliations:** ^1^Department of Anesthesiology, Tohoku University Hospital, Seiryo-cho, Aoba-ku, Sendai, Miyagi, Japan; ^2^Department of Physiology, Tohoku University Graduate School of Medicine, Seiryo-cho, Aoba-ku, Sendai, Miyagi, Japan; ^3^Miyagi University, School of Nursing, Gakuen, Taiwa-cho, Kurokawa-gun, Miyagi, Japan

## Abstract

**Background/Aims:**

Voltage-dependent potassium channels (Kv1.3) are predominantly expressed in lymphocyte plasma membranes. These channels are critical for the activation and proliferation of lymphocytes. Since second-generation antihistamines are lipophilic and exert immunomodulatory effects, they are thought to affect the lymphocyte Kv1.3-channel currents.

**Methods:**

Using the patch-clamp whole-cell recording technique in murine thymocytes, we tested the effects of second-generation antihistamines, such as cetirizine, fexofenadine, azelastine, and terfenadine, on the channel currents and the membrane capacitance.

**Results:**

These drugs suppressed the peak and the pulse-end currents of the channels, although the effects of azelastine and terfenadine on the peak currents were more marked than those of cetirizine and fexofenadine. Both azelastine and terfenadine significantly lowered the membrane capacitance. Since these drugs did not affect the process of endocytosis in lymphocytes, they were thought to have interacted directly with the plasma membranes.

**Conclusions:**

Our study revealed for the first time that second-generation antihistamines, including cetirizine, fexofenadine, azelastine, and terfenadine, exert suppressive effects on lymphocyte Kv1.3-channels. The efficacy of these drugs may be related to their immunomodulatory mechanisms that reduce the synthesis of inflammatory cytokine.

## 1. Introduction

Among antiallergic drugs, second-generation histamine H1 receptor antagonists, such as fexofenadine, cetirizine, terfenadine, and azelastine, are widely used in the treatment of allergic disorders, such as allergic conjunctivitis, chronic rhinitis, urticaria, and asthma [1–3]. They differ from first-generation antihistamines in their higher selectivity for peripheral H1 receptors but lower affinity for H1 receptors in the central nervous system [3]. In addition to their antiallergic properties, second-generation antihistamines exert immunomodulatory properties by actually suppressing the proinflammatory cytokine production from T-lymphocytes [4–8]. Patch-clamp studies revealed that delayed rectifier K^+^-channels (Kv1.3) are predominantly expressed in lymphocyte plasma membranes [9] and that these channels are critical for the initiation of the immune reaction [10–12]. Recently, using murine thymocytes, we revealed drugs, including calcium channel blockers, macrolide antibiotics, and statins, suppressed Kv1.3-currents, and exerted immunomodulatory properties [13–16]. Based on our results, in suppressing the channel currents, these lipophilic drugs appear to generate microscopic changes in the membrane surface structure and thus collapsed the channels conformationally. Among second-generation antihistamines that are more lipophilic than the first-generation ones [17, 18], azelastine and terfenadine have relatively higher lipophilicity [19–21]. Therefore, they were more likely to directly disrupt the thymocyte membranes and thereby suppress the Kv1.3-channel currents. To reveal this, using the patch-clamp whole-cell recording technique in T-lymphocytes (murine thymocytes), we compared the effects of second-generation antihistamines, such as cetirizine, fexofenadine, azelastine, and terfenadine, on the channel currents and membrane capacitance. Here, we show for the first time that these drugs inhibit lymphocyte Kv1.3-channels. We additionally show that the efficacy of azelastine and terfenadine occurred through interactions of the drugs with cellular membranes, which was monitored electrophysiologically by the decreased membrane capacitance.

RETRACTED

## 2. Materials and Methods

### 2.1. Cell Sources and Preparation

Four- to 5-week old male* ddy* mice were purchased from Japan SLC Inc. (Shizuoka, Japan). Mice were anaesthetized deeply using isoflurane. They were sacrificed by dislocating the cervical spine. The Animal Care and Use Committee of Tohoku University Graduate School of Medicine approved our protocol for the use of animals. As we previously described, [13, 15, 16, 22, 23], we separated thymocytes from mouse thymus and resuspended them in external solution containing 145 mM NaCl, 4.0 mM KCl, 1.0 mM CaCl_2_, 2.0 mM MgCl_2_, 5.0 mM Hepes, and 0.01% bovine serum albumin, adjusted with pH 7.2 by titrating NaOH. We kept the isolated cells at room temperature (22-24°C) to use in 4 hours.

### 2.2. Electrical Setup and Patch-Clamp Recordings

Using an EPC-9 patch-clamp amplifier system (HEKA Electronics, Lambrecht, Germany), standard whole-cell patch-clamp recordings were conducted [13, 15, 16, 22, 23]. The patch pipette resistance was maintained 4-6 MΩ when filled with internal (patch pipette) solution containing (in mM): KCl, 145; MgCl_2_, 1.0; EGTA, 10; Hepes, 5.0 (pH 7.2 adjusted with KOH). After we formed a giga-seal, suction was applied briefly to the pipette to rupture the patch membrane. We maintained the series resistance of the whole-cell recordings below 10 MΩ during the experiments. We normalized peak and pulse-end currents by the membrane capacitance, which were expressed as the current densities (pA/pF). All experiments were carried out at room temperature.

RETRACTED

### 2.3. Drug Delivery

We purchased cetirizine dihydrochloride and azelastine hydrochloride, from Tokyo Chemical Industry Co., Ltd. (Tokyo, Japan), and fexofenadine hydrochloride from LKT Laboratories, Inc. (St. Paul, Min., USA). We separately dissolved these drugs in the external solutions to make the final concentration of 100 *μ*M. Terfenadine from Tocris Bioscience (Minneapolis, MN, USA) was dissolved at 10 *μ*M. We delivered one of the drugs to the cells by the standing hydrostatic pressure of 3 cmH_2_O from a nearby pipette, as described previously [13, 15, 16, 22, 23]. Then, we recorded whole-cell membrane currents before and after 30 s exposure to the drugs. To eliminate the possibility that the observed effects were derived from the procedure alone, the external solution was simply applied to the cells and the absence of any significant changes in the channel currents was confirmed.

### 2.4. Membrane Capacitance Measurements

We used the Lock-in amplifier within the EPC-9 Pulse program and employed a sine plus DC protocol [13, 15, 16, 23]. Thus, we monitored the thymocytes' membrane capacitance. We superimposed an 800-Hz sinusoidal command voltage by holding the membrane potential with -80 mV. We continuously recorded the membrane capacitance (Cm), membrane conductance (Gm) and series conductance (Gs), before and after exposing to the drugs for 30 s during the whole-cell patch-clamp recording. Mathematically, we calculate a whole-cell Cm from a parallel-plate capacitor formula:* Cm = εA/d*, where *ε* indicates the dielectric modulus of the plasma membrane;* A* indicates the membrane surface area; and *d* indicates the membrane thickness [24]. Under a physiological condition where* ε* and *d* are almost constant, the changes in Cm are attributable to the alteration in the membrane surface area (*A*) [25].

### 2.5. Electron Microscopy

We fixed the thymocytes, incubated in the external solutions containing no drug, 100 *μ*M azelastine, or 10 *μ*M terfenadine for 10 min, with 4% paraformaldehyde and 3% glutaraldehyde in 0.1 M cacodylate buffer, pH 7.4 for 2 hours at room temperature. After trimming, the specimen was cut into small pieces, postfixed in 1% osmium tetroxide for 1 hour at 4°C, rinsed in PBS, dehydrated in a graded series of alcohol and propylene oxide, and finally embedded in epoxy resin. We prepared ultrathin (80 nm) sections on an ultramicrotome (Ultracut R, Leica, Heerbrugg, Switzerland) with a diamond knife. Then we stained with uranyl acetate and lead citrate and viewed using an electron microscope (JEM-1200, JOEL, Tokyo, Japan).

RETRACTED

### 2.6. Statistical Analyses

We used an EPC-9 amplifier and PulseFit software (HEKA Electronics, Lambrecht, Germany), IGOR Pro 6.2 (WaveMetrics, Lake Oswego, Oreg., USA), and Microsoft Excel 2013 (Microsoft Corporation, Redmond, Wash., USA). Then we analyzed the data and expressed them as means ± SEM. We employed two-way ANOVA and Student's or Dunnett's *t* test, assessing whether they were statistically significant. We considered a p-value < 0.05 being significant.

## 3. Results

### 3.1. Effects of Cetirizine, Fexofenadine, Azelastine, and Terfenadine on Kv1.3-Channel Currents in Murine Thymocytes

To examine the effects of the second-generation antihistamines on Kv1.3- channel currents, we applied external solutions including either 100 *μ*M cetirizine, 100 *μ*M fexofenadine, 100 *μ*M azelastine, or 10 *μ*M terfenadine, to the thymocytes and monitored the changes in the whole-cell currents (Figures 1(a) and 1(b)). When orally administered in humans, the serum concentrations of these drugs are usually below 1 *μ*M under a physiological condition [26–29]. Nevertheless, in some* in vitro* studies, isolated cells, such as cardiomyocytes, needed much higher concentrations of these drugs, including 10 *μ*M terfenadine and as high as 100 *μ*M cetirizine, 100 *μ*M fexofenadine, and 100 *μ*M azelastine, to effectively elicit their inhibitory properties on cardiac K^+^- or Ca^2+^-channel currents [30–33]. In those studies, we dissolved the drugs in the liquid cultured media in advance or persistently injected into the chamber. In our study, however, because the drugs were applied by a puff application method, the exposure of drugs to the cells could be partial or insufficient. To overcome such issues, we applied the drugs to the isolated thymocytes at higher concentrations than those in physiological condition [26–29], such as 100 *μ*M cetirizine, 100 *μ*M fexofenadine, 100 *μ*M azelastine, or 10 *μ*M terfenadine, which were prepared into the patch-pipettes.

Step-like alterations of the membrane potential, from -80 mV (holding potential) to the various levels of depolarizing potential, generated membrane currents in the thymocytes (Figure 1). These currents represented voltage-dependent activation and inactivation patterns that are identical to Kv1.3 [22]. In our previous study, we actually demonstrated in murine thymocytes that margatoxin, a selective inhibitor of the channel, totally inhibited the channel currents [22]. Cetirizine and fexofenadine did not significantly affect the peak Kv1.3-channel currents in thymocytes at the highest voltage-step of + 80 mV (cetirizine: from 266 ± 28.5 to 260 ± 23.7 pA/pF,* n *= 16, Figure 1(a)(B); fexofenadine: from 363 ± 62.3 to 357 ± 62.7 pA/pF,* n *= 13, Figure 1(b)(B)). These drugs rather tended to enhance the peak currents at the lower voltage-steps (Figures 1(a)(A) and 1(b)(A)). However, both cetirizine and fexofenadine significantly lowered the pulse-end currents as demonstrated by the significant decrease in the amplitudes (cetirizine: from 154 ± 18.3 to 107 ± 11.7 pA/pF,* n* = 16,* p* < 0.05, Figure 1(a)(C); fexofenadine: from 228 ± 39.4 to 163 ± 35.6 pA/pF,* n *= 13,* p* < 0.05, Figure 1(b)(C)). Azelastine and terfenadine inhibited the Kv1.3 channel currents in the thymocytes (Figures 2(a)(A) and 2(b)(A)). However, compared to cetirizine or fexofenadine (Figure 1), the peak currents were more dramatically inhibited (azelastine: from 137 ± 24.4 to 67.0 ± 18.4 pA/pF,* n *= 12,* p* < 0.05, Figure 2(a)(B); terfenadine: from 189 ± 39.7 to 117 ± 31.2 pA/pF,* n *= 9,* p* < 0.05, Figure 2(b)(B)) and the pulse-end currents were almost completely suppressed (azelastine: from 101 ± 16.2 to 14.9 ± 4.4 pA/pF,* n *= 12,* p* < 0.05, Figure 2(a)(C); terfenadine: from 114 ± 30 to 34.0 ± 14.7 pA/pF,* n *= 9,* p* < 0.05, Figure 2(b)(C)).

RETRACTED

### 3.2. Effects of Cetirizine, Fexofenadine, Azelastine, and Terfenadine on the Inactivation of Kv1.3-Channel Currents

“Inactivation” is the closing tendency of voltage-dependent ion channels responding to prolonged voltage stimuli after “activation”. Recent advances in molecular biology regarding voltage-dependent* Shaker* family K^+^-channels revealed the presence of two types of inactivation pattern: N-type and C-type [34]. Although the mechanisms are not fully understood, “N-type inactivation” is referred to as the “fast” inactivation, while “C-type inactivation” is as the “slow” inactivation. According to the existing biophysical and mutational evidence [35, 36], N-type inactivation, conferred by a “ball and chain mechanism” involves a blockade of the intracellular mouth of the pore by the partial binding of the extreme N-terminal residues. In contrast, C-type inactivation involves an alteration of residues in the conserved core domain, which leads to the closing of the external mouth.

In the present study, to make the degree of the current inactivation influenced by the second-generation antihistamines more evident, the ratio of the pulse-end currents, which were considered as a “steady-state” currents (*Iss*), to the peak currents (*Ip*) was additionally calculated (Figure 3). Cetirizine and fexofenadine significantly lowered the* Iss/Ip* ratio (Figures 3(a) and 3(b)), indicating that the drugs facilitated the process of inactivation. In contrast, azelastine and terfenadine did not significantly affected the Iss/Ip ratio (Figures 3(c) and 3(d)), suggesting that the drugs inactivated the currents more slowly than cetirizine and fexofenadine did.

RETRACTED

### 3.3. Effects of Cetirizine, Fexofenadine, Azelastine, and Terfenadine on Whole-Cell Membrane Capacitance in Murine Thymocytes

From our results, cetirizine and fexofenadine facilitated the inactivation of the currents faster than that before the application of drugs (Figures 3(a) and 3(b)). According to kinetic studies [34], the results indicated the “N-type inactivation” current patterns, suggesting that these drugs plugged into the open-pores of the channel, inhibiting the currents. In contrast, both azelastine and terfenadine inactivated the currents more slowly than cetirizine and fexofenadine did (Figures 3(c) and 3(d)). These indicated the “C-type inactivation” patterns according to the kinetic studies [34] and suggested that the drugs conformationally collapsed the inactivation gates (selectivity filters) of the pore-forming domains within the potassium channels [22]. Regarding such pharmacological efficacy, azelastine and terfenadine are likely to change the structure of lymphocyte plasma membranes [16]. Using thymocytes, we precisely detected microscopic changes of the cellular membrane surface by measuring the whole-cell membrane capacitance (Cm) [16, 23]. Thus, we employed this electrophysiological technique in the present study to detect the structural changes induced by the drugs within the thymocyte plasma membranes (Figure 4).  Table 1 summarizes the numerical changes in the parameters. When the external solution was simply applied to thymocytes, it did not cause any significant changes in the Cm or other parameters, including the membrane conductance (Gm) and series conductance (Gs) (Table 1). This confirmed the technical precision of our procedure with a puff application of the reagents by a constant hydrostatic pressure using a nearby pipette. The inclusion of 100 *μ*M cetirizine or 100 *μ*M fexofenadine in the patch-pipettes did not significantly alter Cm and other parameters (Figures 4(a) and 4(b); Table 1). However, inclusion of either 100 *μ*M azelastine or 10 *μ*M terfenadine in the patch-pipettes caused significant decreases in the Cm immediately after the drugs were applied (Figures 4(c) and 4(d); Table 1). From these results, azelastine and terfenadine were thought to actually cause the microscopic changes of the structure within the thymocyte membranes. Since the cessation of these drugs during the observation period did not reverse the decreases in the Cm (Figures 4(c) and 4(d); Table 1), the drugs were thought to induce persistent changes in the thymocyte membrane structures.

RETRACTED

### 3.4. Effects of Azelastine and Terfenadine on the Size of Thymocytes and Endocytosis

In T-lymphocytes, membrane trafficking as a result of endocytosis is an important process that regulates the surface expression of membrane proteins, such as T cell receptors [37]. For their recycling, endocytosis constitutively occurs in T-lymphocytes to modulate their immune response [38, 39]. In previous patch-clamp studies, the process of endocytosis in lymphocytes was well monitored by the continuous decrease in the Cm [40, 41]. In our results, since both azelastine and terfenadine significantly decreased the Cm in thymocytes (Figure 4; Table 1), we examined their effects on endocytosis by electron microscopy (Figure 5). At lower magnification, these drugs did not apparently affect the total size of the thymocytes (Figures 5(a)(A), 5(b)(A), 5(c)(A), and 5(d)). At higher magnification of the thymocytes incubated in the external solution alone (Figure 5(a)(B)), there were a few small vesicles in the cytoplasm (arrows) and indentations on the membrane surface (arrow heads), indicating the ongoing process of endocytosis. In thymocytes incubated in azelastine or terfenadine-containing solutions (Figures 5(b)(B) and 5(c)(B)), similar small vesicles were observed in the cytoplasm (arrows). Statistically, there were no significant differences in the total numbers of small vesicles and membrane indentations between thymocytes incubated in the external solution alone and those incubated in the drug-containing solutions (Figure 5(e)). These findings suggested that neither azelastine nor terfenadine affected the process of endocytosis in thymocytes.

## 4. Discussion

In recent studies, second-generation antihistamines were demonstrated to exert immunomodulatory effects by functionally suppressing human leukocytes when they produce proinflammatory cytokines [4–8]. In our study, we demonstrated for the first time that these drugs, which generally antagonize the histamine H1 receptors, additionally suppress the thymocyte Kv1.3-channel currents. By using specific inhibitors of the channel, patch-clamp studies revealed that the Kv1.3-channels are critical for promoting calcium influx and trigger the proliferation and activation of lymphocytes [42–44]. Regarding the molecular mechanisms that are involved, the increased concentration of the intracellular calcium activates the phosphatase calcineurin, which subsequently dephosphorylates the nuclear factor of activated T cells (NFAT), leading to its accumulation in the nucleus and binding to the promoter region of the interleukin 2 (IL-2)-encoding gene [12]. In previous* in vitro* studies, the Kv1.3-channel inhibition by highly selective channel blockers, including ShK-Dap^22^ and margatoxin, was well correlated with the decreased IL-2 production from lymphocytes [9, 45]. Therefore, from our results, the immunosuppressive properties of the second-generation antihistamines are thought to be due to their inhibitory effects on the Kv1.3-channel currents. Our hypothesis is that the second-generation antihistamines' suppression on this delayed rectifier K^+^-channel currents may be involved in the control of cytokines secretion by lymphocytes in inflammatory diseases treated with these drugs in the clinical practice. However, more studies are necessary to calculate that the concentrations of antihistamines used in our study were similar to those obtained in the plasma serum by the use of these same antihistamines on the therapy clinical practice.

RETRACTED

From our results, in contrast to cetirizine and fexofenadine, which failed to affect the peak amplitude of the Kv1.3-channel currents (Figures 1(a) and 1(b)), azelastine and terfenadine significantly inhibited the currents (Figures 2(a) and 2(b)). In our previous study, the amplitude of peak currents was deeply related to the “activation” of the Kv1.3-channel currents, although kinetic studies are necessary to confirm this [22]. In this context, at the lower voltage-steps, cetirizine and fexofenadine may have stimulated the opening of the activation gates of the channels, as we previously demonstrated with chloroquine [22]. In contrast, our results suggested that azelastine and terfenadine were more likely to cause membrane depolarization in thymocytes than cetirizine or fexofenadine. The membrane depolarization undermines the Ca^2+^ flux into the cytoplasm, causing a marked decrease in cellular immunity. This may contribute to the stronger immunosuppressive potency of azelastine and terfenadine than the other second-generation antihistamines, as actually revealed by the decreased production of inflammatory cytokines [6–8].

To reveal the mechanisms of drug-induced prolongation of QT intervals on electrocardiograms, previous studies examined the effects of second-generation antihistamines on various ion channels expressed in cardiomyocytes [18]. In patch-clamp studies using isolated cardiomyocytes or transfected cultured cells, second-generation antihistamines, including cetirizine, fexofenadine, azelastine, and terfenadine, all suppressed the currents of delayed rectifier K^+^-channels, such as Kv1.5 or Kv11.1, which is codified by the human ether-a-go-go related gene (*hERG*) [31, 33, 46, 47]. In these studies, azelastine and terfenadine more potently inhibited the Kv11.1 than cetirizine and fexofenadine did. Kv11.1 is responsible for the cardiac repolarizing K^+^ currents and both azelastine and terfenadine actually increased the action potential duration of cardiomyocytes [33, 48]. Therefore, the blockade of this channel was considered to be the primary mechanism by which azelastine and terfenadine cause QT interval prolongation.

RETRACTED

Mathematically, we calculate a whole-cell Cm from a parallel-plate capacitor formula:* Cm = εA/d*, where* ε* indicates the dielectric modulus of the plasma membrane;* A* indicates the membrane surface area; and *d* indicates the membrane thickness [24]. Under a physiological condition where* ε* and *d* are almost constant, the changes in Cm are attributable to the alteration in the membrane surface area (*A*) [25]. Therefore, we frequently measured the Cm to monitor the process of exocytosis in secretory cells or endocytosis in phagocytic cells, in which the total membrane surface area is gradually increased or decreased [40, 41, 49–52]. In the present study, however, despite the decrease in the Cm (Figures 4(c) and 4(d)), neither azelastine nor terfenadine apparently affected the size of the thymocytes (Figures 5(a)(A), 5(b)(A), 5(c)(A), and 5(d)), nor did they affect the process of endocytosis in the cells (Figures 5(a)(B), 5(b)(B), 5(c)(B), and 5(e)), indicating that “*A*” remained constant in the formula after the drug application. In such a condition, the increase in *d* was likely to be primarily responsible for the decreased Cm [12]. Generally, first-generation antihistamines are more lipophilic than second-generation antihistamines [17]. Among second-generation antihistamines, since azelastine and terfenadine are relatively more lipophilic than the others [19–21], they were thought to distribute more freely into the lipid bilayers of the plasma membranes. Thus, the decrease in the Cm was considered to be mainly attributable to the increased membrane thickness (*d*) caused by the drug-membrane interactions [53]. Then, from inside the membranes, the drugs may directly intrude into the composite domains of the channels, constricting or conformationally collapsing the selectivity filters of the pore-forming domains within the channel [34]. Consequently, azelastine and terfenadine were thought to induce “C-type inactivation” of the Kv1.3-channel currents (Figures 2 and 3).

According to our previous animal studies, Kv1.3-channels were overexpressed in lymphocytes and were pathologically responsible for their* in situ* proliferation within kidneys and the deterioration of renal fibrosis [54]. We further revealed that benidipine, one of the dihydropyridine calcium channel blockers (CCBs), actually improved the progression of renal fibrosis [54] by strongly inhibiting the lymphocyte Kv1.3-channels [13]. Recently, targeting the channels, we suggested novel pharmacological approaches in the treatment of “chronic inflammatory diseases”, including chronic kidney disease (CKD), chronic obstructive pulmonary disease (COPD), and inflammatory bowel disease (IBD) [55–57]. From our results, similar to CCBs, statins and macrolide antibiotics [13–16], second-generation antihistamines, such as cetirizine, fexofenadine, azelastine, and terfenadine, also efficiently suppressed the Kv1.3-channel currents in thymocytes (Figures 1 and 2). Therefore, these drugs may be additively used as potent inhibitors of “chronic inflammatory diseases”.

RETRACTED

## 5. Conclusion

In conclusion, this study revealed for the first time that second-generation antihistamines, including cetirizine, fexofenadine, azelastine, and terfenadine, inhibit the Kv1.3-channel currents in lymphocytes. Of note, azelastine and terfenadine significantly lowered the membrane capacitance. Since these drugs did not affect the process of endocytosis in lymphocytes, they were thought to have interacted directly with the plasma membranes. Such efficacy of these drugs may be related to their immunomodulatory mechanisms by which they reduce the inflammatory cytokine synthesis.

## Figures and Tables

**Figure 1:** *Effects of cetirizine and fexofenadine on Kv1.3 channel currents in murine thymocytes*. The effects of 100 *μ*M cetirizine (a) and 100 *μ*M fexofenadine (b). (A) Typical whole-cell current traces at different voltage-steps recorded before and after the application of either drug. The currents were elicited by voltage-steps from the holding potential of -80 mV to -40, 0, 40, and 80 mV, as depicted in the voltage protocol. Each pulse was applied for a 200-ms duration between 10-second intervals. (B) Peak current densities (peak currents normalized by the membrane capacitance) obtained from the records in (A) at the voltage-step of 80 mV. (C) Pulse-end current densities (pulse-end currents normalized by the membrane capacitance) obtained from the records in (A) at the voltage-step of 80 mV. ^**#**^* p* < 0.05* vs.* before the drug application. Values are means ± SEM (cetirizine,* n* = 16; fexofenadine,* n* = 13). Differences were analyzed by ANOVA followed by Dunnett's or Student's *t* test.

**Figure 2:** *Effects of azelastine and terfenadine on Kv1.3 channel currents in murine thymocytes*. The effects of 100 *μ*M azelastine (a) and 10 *μ*M terfenadine (b). (A) Typical whole-cell current traces at different voltage-steps recorded before and after the application of either drug. The currents were elicited by voltage-steps from the holding potential of -80 mV to -40, 0, 40, and 80 mV, as depicted in the voltage protocol. Each pulse was applied for a 200-ms duration between 10-second intervals. (B) Peak current densities (peak currents normalized by the membrane capacitance) obtained from the records in (A) at the voltage-step of 80 mV. (C) Pulse-end current densities (pulse-end currents normalized by the membrane capacitance) obtained from the records in (A) at the voltage-step of 80 mV. ^**#**^* p* < 0.05* vs.* before the drug application. Values are means ± SEM (azelastine,* n* = 12; terfenadine,* n* = 9). Differences were analyzed by ANOVA followed by Dunnett's or Student's *t* test.

RETRACTED

**Figure 3:** *Effects of second-generation antihistamines on the degree of inactivation of Kv1.3 channel currents*. The effects of 100 *μ*M cetirizine (a), 100 *μ*M fexofenadine (b), 100 *μ*M azelastine (c), and 10 *μ*M terfenadine (d) on the ratio of the pulse-end currents, which were considered as a “steady-state” currents (*Iss*), to the peak currents (*Ip*) obtained from the current traces at the voltage-step of 80 mV. ^**#**^* p* < 0.05* vs.* before the drug application. Values are means ± SEM (cetirizine,* n* = 5; fexofenadine,* n* = 5; azelastine,* n* = 5; terfenadine,* n* = 4). Differences were analyzed by ANOVA followed by Dunnett's or Student's *t* test.

**Figure 4:** *Second-generation antihistamines-induced changes in thymocyte membrane capacitance, series, and membrane conductance*. After establishing the whole-cell configuration, external solutions containing 100 *μ*M cetirizine (a), 100 *μ*M fexofenadine (b), 100 *μ*M azelastine (c), or 10 *μ*M terfenadine (d) were delivered for 30 sec to single thymocytes. Membrane capacitance, series, and membrane conductance were monitored for at least 2 min. Cm, membrane capacitance; Gs, series conductance; Gm, membrane conductance.

**Figure 5:** *Electron microscopic images of thymocytes after incubation in azelastine or terfenadine*. Thin-section electron micrographs of thymocyte membrane surface after incubating the cells in the external solutions containing no drug (a), 100 *μ*M azelastine (b) or 10 *μ*M terfenadine (c). Low-power (A) and high-power (B) views. (d) Diameters of thymocytes incubated in each solution were measured and averaged. (e) Endocytosis was quantified in thymocytes incubated in each solution by counting the numbers of small vesicles in the cytoplasm (arrows) and indentations (arrow heads) on the membrane surface per cells. Values are means ± SEM (*n* = 20). Differences were analyzed by ANOVA followed by Dunnett's or Student's *t* test.

RETRACTED

**Table 1:** Summary of changes in membrane capacitance after application of cetirizine, fexofenadine, azelastine, and terfenadine.

Agents	*n*	*Cm* before drug application	*Cm* after drug application	*ΔCm (fF)*
		(pF)	(pF)	
External Solution	6	3.48 ± 0.30	3.41 ± 0.29	70.0 ± 29.1
100 *μ*M Cetirizine	5	2.66 ± 0.28	2.61 ± 0.27	86.0 ± 11.2
100 *μ*M Fexofenadine	6	3.41 ± 0.43	3.36 ± 0.44	65.0 ± 14.8
100 *μ*M Azelastine	6	4.34 ± 0.73	3.63 ± 0.54^*♯*^	706 ± 228
10 *μ*M Terfenadine	5	2.93 ± 0.42	2.67 ± 0.39^*♯*^	267 ± 74.4

Values are means ± SEM. *Cm* = membrane capacitance.

^#^ *p* < 0.05 *vs*. Cm before drug application.

## Data Availability

The data used to support the findings of this study are available from the corresponding author upon request.
